The article "Exploring Multiple Application Scenarios of Visual Communication Course Using Deep Learning Under the Digital Twins" was published in 2022. Journal: Comput Intell Neurosci.

# Exploring Multiple Application Scenarios of Visual Communication Course Using Deep Learning Under the Digital Twins

**DOI:** 10.1155/2022/5844290

**Published:** 2022-02-15

**Authors:** Guan-Chen Liu, Chih-Hsiang Ko

**Affiliations:** ^1^Department of Design, National Taiwan University of Science and Technology, Taipei, Taiwan; ^2^Visual Communication Design, Jinwen University of Science & Technology, New Taipei City, Taiwan

## Abstract

The emergence of intelligent technology has brought a particular impact and allows for virtuality-reality interaction in the educational field. In particular, digital twins (DTs) feature virtuality-reality symbiosis, solid virtual simulation, and high real-time interaction. It has also seen extended applications to the field of education. This study optimizes the design of the visual communication (Viscom) course based on the deep learning (DL) algorithm. Firstly, the theory of DL is analyzed following the relevant literature, and the typical DL networks, network structures, and related algorithms are introduced. Secondly, Viscom technology is expounded, and DL technology is applied to the Viscom course. Then, the applicability and feasibility of DL in the Viscom course are analyzed through a questionnaire survey (QS) design by collecting students' attitudes towards Viscom courses before and after the experiment. After introducing DL into the Viscom course, the results show that students' learning interest and satisfaction with the practical knowledge mastery have increased. However, the satisfaction with theoretical knowledge mastery before practical courses has decreased; overall, the teaching effect of the Viscom course has been improved. Therefore, the introduction of DL into the DT-enabled Viscom can provide a reference for developing the Viscom course. The research content offers technical support (TS) for integrating DT technology and modern education.

## 1. Introduction

With the popularization of artificial intelligence (AI), big data analytics (BDA), fifth-generation (5G) communication, and Internet-of-things (IoT) technology, intelligent technologies are seeing diverse application scenarios in different industries. In particular, digital twins (DTs) are a product life cycle (PLC)-oriented management tool driven by model information flow. Its core is the process of data collection, aggregation, analysis, and decision-making (DM), which provides technical support (TS) and data basis for future production and construction. It is now possible to apply DT technology to construct a personalized education environment, realize the forward-looking research of mixing virtuality and reality, and build a novel, brilliant, and intelligent education model. Visual communication (Viscom) is the inevitable product of the development of the times. Adjusting the Viscom course to promote students' learning has become the primary concern in the research and educational field. On the other hand, deep learning (DL) is a novel research algorithm. Applying DL to Viscom courses can improve teaching efficiency and bring more diversified and complex visual information [1]. The present work adopts DL based on the unique features of the DL algorithms. The ultimate goal of DL is to empower the machine to analyze and learn like human beings and recognize text, image, sound, and other data, far surpassing the previous relevant technologies. Remarkably, applying DL to Viscom courses can vividly impart boring theoretical knowledge and arouse students' classroom enthusiasm.

DTs are a dynamic high simulation digital model under specific closed-loop data and driven by directional multidimensional heterogeneous data. It can provide active or responsive services to particular objects in different situations for Chinese vocational education and training (VET), thereby establishing more professional VET models [2]. Significantly, Viscom design will achieve more intellectual development under the collaborative efforts of various emerging technologies. Compared with the shallow network model, the multilayer neural network (NN) model includes more complex functions and more robust feature learning and expression ability. Therefore, DL has broad application prospects. Introducing DL technology can help break through the limitations of traditional Viscom courses, improve the course flexibility, and expand the innovative ideas and space of Viscom courses under the background of DTs.

Fan et al. [3] thought that the way of Viscom was full of modern life. They designed a reference game based on drawing, finding that people could communicate more effectively by sharing information; in other words, the players away from the specific target could get better recognition using less depiction. Garland et al. [4] applied the DL generative confrontation network (GAN) to micro-vision and constructed the micro-vision GAN model based on DL; the results of simulation and analysis found that the constructed model presented high accuracy in feature extraction (FE). Zhu et al. [5] did a comprehensive review of audiovisual (AV) learning and found that the essence of AV learning was to utilize the relationship between AV patterns. Meanwhile, AV learning made rapid progress with the rapid development of DL. They subdivided the AV learning tasks, discussed the remaining challenges in each subarea separately, and summarized their data sets. In summary, scholars and researchers have put forward diverse theoretical views and research methods on DL algorithms and Viscom from different angles. The present work draws lessons from and optimizes upon these methods. The purpose is to apply the novel DL algorithms to Viscom courses from the overall point of view. Kamilaris et al. [6] compared and analyzed the conceptual connotation of DL and DTs from the perspective of educational technology (ETEC) in the understanding of deep learning. They believed that both technologies were necessary for learning. In particular, DL was learning declarative, procedural, and strategic knowledge. DL paid more attention to reconstructing learners' cognitive structure, and DL and DTs were correlated and overlapped. Then, they also analyzed the connotation and implementation of DL technology.

The above literature review suggests that the research on DL and Viscom course has made some progress, but there is little research on the integration of DL into the Viscom course under the background of DTs. Thereupon, this study first expounds on the relevant theories of DL and Viscom and then systematically discusses the development process of the Viscom course and the influence of DL technology in the Viscom course. Afterward, the application effect of DL in the Viscom course is investigated by questionnaire survey (QS). Further, the practicability and feasibility are analyzed for the proposed DL-based Viscom course under the background of DTs. Finally, the research deficiencies are summarized, and relevant suggestions are put forward to develop the Viscom course. Innovatively, based on DL's theoretical and technical framework, DL technology is introduced into the construction of the Viscom course, and the new development model of future education is explored under the background of DTs.

## 2. DL Algorithm and Viscom Course

Viscom design is expressed and communicated to the audience through visual media, which embodies the characteristics of the times, graphic design, and rich connotation. Information obtained during the learning process by applying the DL algorithm to Viscom can significantly facilitate the interpretation of data, such as text, image, and sound. Its ultimate goal is to empower the machine to analyze and learn like human beings to recognize characters, images, sounds, and other data. Therefore, DL can make Viscom more vivid. In turn, Viscom can enrich the research field of DL.

### 2.1. DL Algorithm

Theoretically, DL is a branch of machine learning (ML) that learns historical data and extracts valuable information. DL algorithm can achieve self-improvement through learning. The network structures of standard DL algorithms include multilayer perceptron (MLP) and convolutional neural network (CNN), both of which require nonlinear activation function (AF) [7–9].

A fully connected multilayer NN structure was divided into three layers: the input layer, the hidden layer (one or multiple layers), and the output layer. Meanwhile, nodes of each layer were connected to each lower layer node.  Figure 1 shows the specific network structure.

The propagation algorithm is expressed as follows:

(1) $$\begin{array}{c} a_{0}=x. \end{array}$$

In equation (1), *x* represents the model input, and *a*_0_ indicates the regularization coefficient.

(2) $$\begin{array}{c} Z_{k}=W_{k}a_{k-1}+b_{k}. \end{array}$$

In equation (2), *Z*_*k*_ represents the input of each layer, *k* indicates the network depth, and *k* ∈ (1, *L*) is an integer. *W*_*k*_ denotes the *k*th layer weight matrix, and *b*_*k*_ denotes the *k*th layer offset vector.

(3) $$\begin{array}{c} a_{k}=f\left(Z_{k}\right). \end{array}$$

In equation (3), *a*_*k*_ represents the *k*th layer output.

(4) $$\begin{array}{c} y^{\prime }=a_{L}. \end{array}$$

In equation (4), *y*′ represents the network output, and *a*_*L*_ denotes the output value of the *L*th layer (the last layer).

(5) $$\begin{array}{c} J=L\left(y{}^{\prime },y\right)+\alpha \phi \left(\theta \right). \end{array}$$

In equation (5), *J* represents the loss function (LF), and *y* stands for the real value corresponding to the input sample. *L*(*y*′, *y*) refers to the difference between the input sample's actual value and the network's output. *ϕ*(*θ*) denotes a regular term added to prevent overfitting, including all parameters *W* and *b* in the model.

(6) $$\begin{array}{c} g⟵\nabla_{Z_{k}}J=g⊙f^{\prime }\left(Z_{k}\right). \end{array}$$

In equation (6), *g*⟵∇_*Z*_*k*__*J* represents the gradient of the LF *J* for the input *Z*_*k*_ of each layer.

(7) $$\begin{array}{c} \nabla_{w_{k}}J=ga_{k-1}^{T}+\alpha \nabla_{w_{k}}\phi \left(\theta \right). \end{array}$$

In equation (7), ∇_*w*_*i*__*J* represents the gradient of *J* concerning the parameter *w*_*k*_ of each layer.

(8) $$\begin{array}{c} \nabla_{b_{k}}J=g+\alpha \nabla_{b_{k}}\phi \left(\theta \right). \end{array}$$

In equation (8), ∇_*b*_*k*__*J* represents the gradient of *J* concerning the parameter *b*_*k*_ of each layer.

Through the LF *J*, the parameters *W* and *b* in the model can be obtained. After the LF gradient is calculated for each layer's parameters, the parameters *W* and *b* of each layer can be updated through the gradient-based optimizer (GBO).

CNN is different from a NN with fully connected layers and includes the input layer, convolution layer, pooling layer (lower sampling layer), fully connected layer, and output layer [10].  Figure 2 displays the network structure.

The specific algorithm is expressed as follows:

(9) $$\begin{array}{c} H_{i}=f\left(H_{i-1}⊗W_{i}+b_{i}\right). \end{array}$$

In equation (9), *H*_*i*_ represents the feature graph of the *i*th layer; ⊗ indicates the convolution operation between the *i* − 1th layer feature graph and the *i*th layer feature graph.

(10) $$\begin{array}{c} H_{i}=\text{subsampling}\left(H_{i-1}\right). \end{array}$$

Equation (10) shows the operation of the pooling layer.

### 2.2. Development of Viscom Course Under the Background of DTs

The term *visual communication* gets popular as early as 1960, at the Tokyo *World Design Conference* in Japan. Initially, all creations expressed through “vision” are referred to as Viscom design. Then, the design of printing art in Europe and America in the 19th century has considerably promoted the development of Viscom. In China, back in the Qing Dynasty (1636–1912), foreign artists have stepped into the Chinese territory to establish schools with Viscom education courses; however, Viscom design therein is limited to Science and Technology (S&T) levels and the times and only involves layout design. With the progress of the times and S&T, mainly the emergence of computer networks (CNETs), people's requirements for Viscom design have improved radically, which, in turn, helps make Viscom design more colorful. Correspondingly, people pay ever-more attention to Viscom education. The introduction of the DL algorithm into the Viscom course is an expansion and promotion of Viscom design education [11].

DT technology is a tool to manage complex information through data visualization. It represents and maximizes the information value of twin objects in model language, thereby providing real-time, efficient, and intelligent service solutions for individuals, organizations, and systems. Viscom design uses human visual symbols to convey information to the receiver. Bridged by specific visual language and media, designers and receivers can communicate and interact more efficiently and freely, ignoring language, age, or skin color while sharing common consensus on things they see [12]. Notably, in the DT-enabled systems, the virtual model parameters can reflect the real-time dynamic information of natural objects over the IoT, BDA, and AI technologies. Through the feedback mode of virtuality-reality interaction, real-time DM is provided for the Viscom course from multidimensional data fusion, realizing the efficient coordination of various stages in the Viscom courses [13].

Through the visual media, the audience can see the era characteristic graphics with rich connotations created by the Viscom designer. With the development of CNETs, Viscom has completely a single to multiple and static to three-dimensional (3D) dynamic transformation. Research shows that visual pathway accounts for more than 60% of normal human information transmission. Therefore, it is imperative to develop the Viscom design course [14]. From commercial art to arts and crafts, and from printing art design to decoration design and today's graphic design, Viscom design, carried upon the visual media, uses visual symbols to express and transmit information. Traditionally, Viscom design is technically called graphic design. With its contemporary development, there is hardly any difference between Viscom design and graphic design, with the same design contents.

Therefore, DT technology emphasizes collecting and interpreting underlying real-time multidimensional data. In contrast, the human-computer interface (HCI) mainly presents the simulation model of physical objects to visually display the progress of the Viscom course through model interaction and visual data. Additionally, DTs feature an interpersonal communication function. Integrating DT and DL technology can provide participants with a more immersive first lesson experience and realize a general VI perception.

### 2.3. DL and Viscom

Nowadays, people are highly dependent on computers and the Internet, and CNETs have become the central information communication channel. Besides, the application of DL in vision is concentrated in computer vision (CV), such as image classification, object detection, image segmentation, target tracking (TT), and 3D reconstruction. This section applies the DL to Viscom courses to conduct relevant research [15].

#### 2.3.1. Image Classification

One of the primary tasks of the CV is image classification. Some physical entities have distinct features and can be easily distinguished. In contrast, others may not be easily distinguishable due to similar or imperceptible features. These undistinguishable entities consume vast amounts of time and complex calculations by both humans and computers. Before introducing DL, computers' object recognition and classification were limited in numbers and types; only those significant features are extracted for object recognition and distinction; computer recognition and classification performance will be significantly reduced when features are not noticeable. With the introduction of DL, computers' image classification ability and image classification accuracy have improved substantially, from 80% to over 95%, much close to the human resolution and far more than 50% before the introduction of DL.

#### 2.3.2. Object Detection

Simply, object detection is to coordinate the specific object or point in an image or video, but in practice, many factors can affect the process, including angle, size, distortion, and background complexity. Similarly, before the introduction of DL, the computer mainly relied on artificial assistance, such as manual designated features; if the manual aid is not in place or the expression is unclear, the computer cannot accurately detect the object. The introduction of DL solves such awkwardness. The appearance of SPPNet and its optimization variants have helped improve the object detection of computers, reaching an astounding 80%.

#### 2.3.3. Image Segmentation

Simply, it distinguishes specific regions where different things exist in an image. According to segmentation accuracy, image segmentation can be divided into semantic segmentation (SS), instance segmentation, and panoramic segmentation. According to the pixel type in the image, the specific category is distinguished based on pixel-level discrimination, and all things in the image, including the background, can be segmented based on the first two categories. Due to their limitations, the current DL algorithms are mainly applied to SS, which is divided into region-based and pixel-based SS. The latter's performance is better than the former.

#### 2.3.4. TT

TT predicts the objects' subsequent position based on its current coordinates. TT is a complex process and is interfered with by many factors, such as scene brightness and background complexity. The traditional tracking method is volatile. At present, the role of DL in TT is not very obvious, but it has shown great potential. If researchers can solve DL's learning difficulty using a single initial location, DL will make a significant breakthrough in TT.

#### 2.3.5. 3D Reconstruction

3D reconstruction is the core of CV research. From basic 3D modeling to the cutting-edge field of intelligent robots, 3D reconstruction is the key method. Before introducing DL, 3D reconstruction was mostly based on geometric principles because it required specific conditions, such as multiple views, so its application is limited to specific environments. After the introduction of CNN, the relevant research on 3D reconstruction has gradually caught up. With more NN structures being introduced, the scene restoration depth of the monocular image is more than doubled.

### 2.4. Viscom Course under the Influence of DL

The above research shows that DL significantly influences Viscom and can promote the development of traditional CV. Further, it intellectualizes Viscom to the human level or over human intellectualization. Meanwhile, DL has a particular impact on the current Viscom courses. The recent Viscom course divides visual problems into three classes: low, medium, and high, which correspond to image enhancement and restoration, image FE, and object recognition and understanding, respectively. Hence, researchers emphasize the hierarchical processing of visual information (VI). Because of the specific node connection pattern and automatic FE, it no longer depends on the hierarchical processing of VI. Therefore, to introduce DL into Viscom courses, there is a need to innovate the current teaching content system [16–20].

First, the basic theory of DL should be introduced into the teaching content to make students fully understand the application mechanism of DL in CV.  Table 1 lists the main knowledge points involved.

In particular, there is a need to introduce a basic network model with significant application value and study the training and optimization methods to understand its principle, concept, and calculation method and avoid fitting failure caused by the lack of basic theory. Then, these basic ideas can innovate the teaching content. Meanwhile, special courses introducing traditional processing methods can be adapted: there is a need to introduce theoretical principles and shorten the content about traditional algorithms [21–23]. The present work focuses on the theory and application of the DL algorithms, including the network selection and optimization and dataset construction. The research results help integrate theory into the curriculum. Further, there is a need to fully utilize the advantages of CNETs to implement online teaching, offline explanation, and teaching design as much as possible to design and explain some experiments. Lastly, actual case analysis can improve the classroom vividness, thereby helping students understand and remember corresponding knowledge points.

### 2.5. Research Method

Literature review method: firstly, China National Knowledge Infrastructure (CNKI), Google Academic, and other channels are used to query data. Secondly, many articles and works are consulted from columnists and relevant Internet information. Besides, many journals and related books from the school library are reviewed, such as *Basic Course of Layout Design* and *Viscom Design Practice.* The collection and summary of the data set provide a solid theoretical basis for the research ideas and methods. Comparative analysis method: it refers to the multiparty comparison of two or more research objects to explore the similarities and differences between them and study and learn from good manners to research how to apply DL algorithms to Viscom courses. QS method: it is a method widely used in social surveys globally. A questionnaire refers to the form used for statistics and surveys to display questions. QS method can measure the research problems through controlled measurement to collect reliable data. For readers and researchers to deeply understand the changes in Viscom experimental teaching before and after the introduction of DL, 300 QSs are randomly distributed to different types of students in November 2020. For the scientificity concern of the QS, the designed QS contents are reviewed by experts from relevant majors before the distribution, and the unreasonable parts in the QS design have been revised accordingly. For recovery rate consideration, face-to-face distribution and on-spot collection are employed. As a result, 270 copies of QSs are recovered, with a recovery rate of about 90%; the number of effective copies is 230, with an effective recovery rate of 85.19%.

Next, the data of the QS are tested by Kaiser–Meyer–Olkin (KMO) coefficient. The following equation expresses the specific calculation:

(11) $$\begin{array}{c} \text{KMO}=\frac{\sum \sum_{i\neq j}r_{ij}^{2}}{\sum \sum_{i\neq j}r_{ij}^{2}+\sum_{i\neq j}r_{ij•1,2...k}^{2}}. \end{array}$$

In equation (11), *r*, *i*, *j*, and *k* represent correlation coefficient (CC), dependent variable, independent variable, and quantity, respectively.  Table 2 signifies the *KMO* measurement criteria.

Based on the relevant statistic knowledge, the data validity of the designed QS is analyzed by SPSS 23. The KMO is calculated as 0.869, 0.8∼0.9, and (*p*=0) <0.01. It shows that the QS data are suitable for factor analysis, and the QS has good validity.

### 2.6. Design of Experiment

Noticeably, the practical course is vivid and straightforward. According to the previous research on students' interest in learning and learning effect, compared with the theoretical classroom course, students prefer practical course, in which the practical link is particularly impressive and has a good teaching effect [24–27]. To this end, there is a need to innovate the teaching content from more practical teaching and design more experimental tasks, such as image denoising, feature detection, semantic SS, object detection and tracking, and stacked auto-encoder (SAE) through the GAN model, full CNN, deep CNN, and RNN model.

Image denoising and image SS are common CV tasks in DL. Then, this section selects five experimental contents and their corresponding network models to facilitate the training and learning of DL networks [28].

Subsequently, the experiment extends the duration of practical teaching appropriately, as shown in Table 3.

Table 3 shows that after the innovation of the Viscom course, the theoretical course time is reduced, and the practical course time is increased. The total teaching time of 50 hours has not changed. More emphasis is put on practical teaching.

Before and after the introduction of DL, the change in Viscom experiment teaching should be one of the key points of the Viscom course. Through in-depth explanation, students can distinguish different algorithms, pay more attention to the characteristics of the Viscom course after the introduction of DL, and focus on the data preprocessing, model design, and parameter optimization of the DL models. The innovative course explains in detail the application principle of DL algorithm, model construction, model training, parameter selection, algorithm optimization, etc., and helps students quickly master the principle and application of DL [1, 4, 29, 30].

The section explicitly studies the image SS based on the CNN structure illustrated in Figure 2 to explore the segmentation model's principle, construction, and training. The samples are chosen from the open data set on the network, programmed with Python, and based on the TensorFlow framework. The experimental processes are as follows:

1. Data Preprocessing: data preprocessing divides data sets into three categories: training, verification, and testing; the numerical values of features are standardized to the same interval for comparison; meanwhile, data preprocessing should adjust image size to be compatible with hardware devices; specific methods should be chosen for data enhancement to avoid data overfitting.
2. Model Construction: The model construction process includes parameter adjustment, such as the number of convolution pooling layers, the number of neurons distributed to each layer, and the volume of the convolution kernel. The existing network structure is usually improved and adjusted according to the needs to facilitate the experiment.
3. The Design of LF: the LF is introduced to measure the difference between the actual input sample and the output. Obviously, the performance of the LF directly affects the performance of the model. In image SS, the pixel classification problem can replace the segmentation problem; that is, the LF reflects the classification accuracy for pixels. Under specific experiments, different LFs can be constructed and compared to find the most suitable model.
4. Model Training: The RNN's training process is challenging because it involves many problems, such as gradient explosion and disappearance. Then, the model training process first initializes the parameters and then optimizes the algorithm. Meanwhile, different parameter setting schemes and algorithms can be combined to observe their adaptability to different models.
5. Comparison Analysis: One of the key points is to compare the Viscom courses before and after the course innovation, thereby evaluating the advantages of introducing the DL algorithm. Therefore, indexes can be selected to evaluate the Viscom course before and after the experiment. In short, this study studies the application of DL to the Viscom course from these five aspects to obtain a more accurate research result. The data preprocessing results and the comparison between before and after the introduction of DL to Viscom courses are in line with the realistic, logical program.

## 3. QS of Students' Attitude Towards Viscom Course Before and After the Introduction of DL

### 3.1. Proportion of Respondents

Subsequently, SPSS 22.0 tests the correlation between the selected QS data.  Table 4 reveals the specific results.

Table 4 shows the relevant test results among students of different grades and students' attitudes towards Viscom courses before and after the introduction of DL. The results show that the CCs among students of different grades are 0.712, 0.5856, and 0.5961, respectively, indicating a positive correlation between them. Similarly, the CCs between students' attitude, interest, and satisfaction with Viscom courses are 0.5269, 0.5697, and 0.6245, respectively, indicating that there is also a positive correlation between them. The CCs between satisfaction and interest of students in different grades are 0.634, 0.6893, and 0.6358, respectively; this indicates that there is also a correlation between them, and the correlation is the highest among the three groups of data. Overall, CC > 0.7 indicates a very close relationship, CC between 0.4 and 0.7 implies a close relationship, and CC between 0.2 and 0.4 shows a general relationship. The factors of selected QS data have a good correlation and can meet the research requirements.

Next, QS was conducted on the teaching effect of the Viscom course with the DL algorithm. Totally, 100 respondents were randomly recruited. The proportion of respondents is shown in Table 5.

This section selects 50 men and 50 women as research subjects to ensure the credibility of the experimental results. Of these, 59.36%, 31.89%, and 8.75% of the respondents are 20–25, 26–30, and 30–35 years old, respectively; 54.6%, 19.6%, 23.7%, and 2.1% of the respondents are undergraduates, junior college students, postgraduates, and doctoral students, respectively.

### 3.2. QS of Students' Interest

Figure 3 presents the QS results of students' interest in Viscom courses before and after the introduction of DL.

Figure 3 displays that 27 people were not interested in the Viscom course before the introduction of DL, and the remaining 73 were interested in the Viscom course. After the introduction of DL, the number of people satisfied with Viscom courses has increased to 92, and only eight people still have no interest in the course. Hence, the introduction of DL can improve the students' interest in Viscom courses.

### 3.3. QS on the Satisfaction of Students' Mastery of Knowledge

Figure 4 manifests the QS results of students' satisfaction with the mastery of theoretical knowledge before the practical course before and after the introduction of DL.

Figure 4 implies that before introducing DL, 54 students were satisfied with their mastery of the corresponding theoretical knowledge before the practical course; 29 students thought they were relatively satisfied, while 17 students were dissatisfied. After introducing DL, the number of students dissatisfied with their mastery of the corresponding theoretical knowledge before the practical course has increased to 21. In contrast, relatively satisfied students have increased to 36, and the number of satisfied students has decreased to 43. Therefore, after compressing the theoretical class hours and prolonging the experimental teaching time, students are more satisfied with the Viscom course. Probably, it is because the theoretical course is boring, and the experimental course can meet students' hands-on operation ability and is more interesting.

Figure 5 draws the QS results of students' satisfaction with the mastery of the practical course before and after the introduction of DL.

Figure 5 suggests that before the introduction of DL, the number of dissatisfied students with their mastery of practical courses was 19, and the number of relatively satisfied students was 42. The number of satisfied students was only 39. After the introduction of DL, the number of dissatisfied students is only 7, the number of relatively satisfied students has not changed much, only two less than before, and the number of satisfied students is over half of the total respondents. Apparently, the voice and image recognition competency in DL technology has also improved students' interest in learning when enriching teaching links.

### 3.4. Research on Comprehensive Teaching Effect

Figure 6 illustrates the QS results of the comprehensive teaching effect of the Viscom course before and after the introduction of DL.

Figure 6 illustrates that before the introduction of DL, as many as 39 students think that the course has no teaching effect, and 24 students think that the teaching effect is perfect. After introducing the DL algorithm, only five people believe that the Viscom course has no effect, and the number of people who think that the teaching effect of the course is perfect has risen to 52. Interestingly, before and after introducing the DL algorithm, the number of students who think that the Viscom course has only limited effect has not changed significantly, just from 37 to 43. The data changes in Figure 6 corroborate that the introduction of DL into the Viscom course has improved students' learning interest, satisfaction, and comprehensive teaching effect, which shows that the traditional Viscom course needs continuous innovation to arouse students' learning interest. In a similar study, Zhu [31] discussed three issues: the educational reform arising from the application of the DL algorithm, the reasons behind the TS on educational reform, and the mechanism to apply the DL algorithm to promote educational reform [31]; it mainly explored how the algorithm affected educational reform and took students at different stages as the research object. By comparison, the present work studies the students' interest, satisfaction, and comprehensive teaching effect of the Viscom course before and after DL's introduction. It then explores how DL affects the Viscom course. Therefore, the comparison analysis indicates that the present work's research content is more in-depth and comprehensive.

### 3.5. Suggestions

Students are the hope of future national development. Solving the problems existing in the teaching process is a complicated issue that every educator must face. This study puts forward corresponding suggestions from the following three aspects: (1) there is a need to constantly update the educational concept of the development of the times. Educators are the “main force” of ideological and political education. Their educational vision always affects their in-depth thinking on teaching and teaching discourse; (2) educators in higher institutions might need more prosperous knowledge literacy and extensive theoretical literacy, as well as to accumulate more practical experiences to set better examples for students and fellow teachers; and (3) it is imperative for teachers to learn to innovate and often absorb the teaching methods and contents of other Viscom courses, constantly add vitality to the classroom, timely introduce the technique of adaptive DL into the teaching of Viscom, and enhance the interaction between students and teachers, thereby establishing stickiness and improving students' academic performance.

## 4. Conclusion

With the continuous development of S&T, DL technology has penetrated various industries. Taking DTs as the research background and DL as the theoretical basis, the present work discusses the application of the DL algorithm in the Viscom course. It mainly draws the following conclusions: (1) the application of the DL algorithm in the Viscom course has good compatibility, and the students' learning interest in the DL-introduced Viscom course is generally improved. (2) The comparison of the teaching effect of the Viscom course before and after the DL introduction unveils that the proposed DL algorithm has certain practicability and effectiveness. (3) The final research results provide a methodological reference for applying DL and DTs in the Viscom course in the future. Still, the article has some limitations in data acquisition, resulting in data analysis deviations. Additionally, DL has not been discussed in the economic investment in the Viscom course. In the follow-up, the benefit evaluation can be carried out according to the specific situation to utilize the proposed technology in relevant management departments to bring schools or teachers a beneficial impact.

## Figures and Tables

**Figure 1:** Structure of fully connected multilayer NN.

**Figure 2:** Structure of CNN.

**Figure 3:** Students' interest in Viscom course before and after introducing DL.

**Figure 4:** Students' satisfaction with the mastery of the corresponding theoretical knowledge before practical course before and after the introduction of DL.

**Figure 5:** Students' satisfaction with the mastery of practical courses before and after the introduction of DL.

**Figure 6:** Comprehensive teaching effect of Viscom course before and after the introduction of the DL.

**Table 1:** Basic theory of DL.

Theory category	Main knowledge points
Model types	Fully connected NN
	CNN
	RNN (recurrent NN)
	Other network models
Training and optimization	Data preprocessing
	Parameter initialization
	Optimization algorithm and standardization
Framework construction	Caffe and PyTorch, etc.

**Table 2:** KMO measurement criteria.

Type	Range of values	Factor analysis is appropriate
KOM value	<0.9	Very much suitable
	0.8∼0.9	Very suitable
	0.7∼0.8	Fit
	0.6∼0.7	Not very suitable
	0.5∼0.6	Barely fit
	>0.5	Unsuited

**Table 3:** Duration of Viscom course.

Viscom course	Total course duration (h)	Theoretical course duration (h)	Practical course duration (h)
Before course innovation	50	24	26
After course innovation	50	20	30

**Table 4:** Relationship between different research variables.

Project	Students of different grades	Satisfaction of students in different grades	Interest level of students in different grades
Students of different grades	0.712^*∗∗*^	0.5856^*∗∗*^	0.5961^*∗∗*^
Satisfaction of students in different grades	0.5269^*∗∗*^	0.5697^*∗∗*^	0.6245^*∗∗*^
Interest level of students in different grades	0.634^*∗∗*^	0.6893^*∗∗*^	0.6358^*∗∗*^

**Table 5:** Specific proportion of respondents.

Type		Number of people	Proportion (%)
Gender	Male	50	50.00
	Female	50	50.00
Total		100	100.00
Age	20∼25	60	59.36%
	26∼30	31	31.89%
	30∼35	9	8.75%
Total		100	100%
Educational background	Junior college	20	19.6%
	Undergraduate	55	54.6%
	Master	23	23.7%
	Doctor	2	2.1%
Total		100	100%

## Data Availability

The data used to support the findings of this study are included within the article.
